# Trimethylamine N-oxide in atherogenesis: impairing endothelial self-repair capacity and enhancing monocyte adhesion

**DOI:** 10.1042/BSR20160244

**Published:** 2017-03-02

**Authors:** GuoHua Ma, Bing Pan, Yue Chen, CaiXia Guo, MingMing Zhao, LeMin Zheng, BuXing Chen

**Affiliations:** 1 Department of Cardiology, Beijing Tian Tan Hospital, Capital Medical University, Beijing 100050, China; 2 Institute of Cardiovascular Sciences and Institute of Systems Biomedicine, School of Basic Medical Sciences, and Key Laboratory of Molecular Cardiovascular Sciences of Ministry of Education, Peking University Health Science Center, Beijing 100191, China; 3 Medical College of Shantou University, Shantou 515041, China

**Keywords:** Atherosclerosis, Endothelial dysfunction, PKC/ NF-κB, TMAO

## Abstract

Several studies have reported a strong association between high plasma level of trimethylamine N-oxide (TMAO) and atherosclerosis development. However, the exact mechanism underlying this correlation is unknown. In the present study, we try to explore the impact of TMAO on endothelial dysfunction. After TMAO treatment, human umbilical vein endothelial cells (HUVECs) showed significant impairment in cellular proliferation and HUVECs-extracellular matrix (ECM) adhesion compared with control. Likewise, TMAO markedly suppressed HUVECs migration in transwell migration assay and wound healing assay. In addition, we found TMAO up-regulated vascular cell adhesion molecule-1 (VCAM-1) expression, promoted monocyte adherence, activated protein kinase C (PKC) and p-NF-κB. Interestingly, TMAO-stimulated VCAM-1 expression and monocyte adherence were diminished by PKC inhibitor. These results demonstrate that TMAO promotes early pathological process of atherosclerosis by accelerating endothelial dysfunction, including decreasing endothelial self-repair and increasing monocyte adhesion. Furthermore, TMAO-induced monocyte adhesion is partly attributable to activation of PKC/NF-κB/VCAM-1.

## Introduction

Cardiovascular disease (CVD) is the major cause of morbidity and mortality worldwide, with growing incidence in developing countries [1,2]. Atherosclerosis is a key contributor to CVD and is characterized by endothelial dysfunction and subendothelial accumulation of lipids [3]. In recent years, an appreciation for the role of trimethylamine N-oxide (TMAO) in CVDs has gained momentum. Plasma TMAO is a metabolite of the dietary lipid phosphatidylcholine. TMAO was initially identified as a predictor of cardiovascular risk using a metabolomics approach in a large, independent, clinical cohort study [4–6]. Elevated TMAO level in patients with heart failure is positively correlated with prognosis and long-term mortality risk [7,8]. Moreover, dietary TMAO was shown to promote up-regulation of multiple macrophage scavenger receptors associated with atherosclerosis and to enhance development of atherosclerotic lesions in mice [6]. The same mechanistic correlation was found in humans [9]. Collectively, these studies provide convincing evidence that TMAO is a strong risk factor for the development of atherosclerosis.

A large body of evidence suggests that endothelial dysfunction is a key variable in the pathogenesis of atherosclerosis [10–12]. In addition, protein kinase C (PKC) plays a pivotal role in mediating endothelial dysfunction [13]. Endothelial dysfunction, as a comprehensive index of the overall CVD risk factor burden includes three main consequences, exposure of adhesion molecules, the activation and aggregation of platelets, and cholesterol accumulation [3]. Up-regulation of cellular adhesion molecules, such as vascular cell adhesion molecule-1 (VCAM-1), intercellular adhesion molecule-1 (ICAM-1) and E-selectin, play an initial role in the formation of atheromatous plaques [3]. Moreover, for endothelial cells (ECs), PKC activation increases adhesion molecules expression, such as VCAM-1, ICAM-1, E-selectin, interleukin (IL)-6, IL-1, and the activation of NADPH oxidase [14,15]. There is convincing evidence demonstrating that PKC activation is involved in endothelial dysfunction and monocytes adhesion to ECs [16]. Furthermore, the activation of NF-κB is a necessary downstream event of enhanced monocyte adhesion [16–21].

Although the association between TMAO plasma levels and atherosclerosis progression is well proven, the exact mechanism of this association is not entirely defined. Given the vital role of endothelial dysfunction in atherosclerotic disease progression, it is tempting to suggest that TMAO promotes atherosclerosis by increasing endothelial dysfunction. The present data suggested a new pathway by which TMAO-induced EC dysfunction and monocyte adhesion to the arterial wall and contributed to atherosclerosis. Our study showed that TMAO caused impaired self-repair and PKC-dependent NF-κB activation, VCAM-1 expression and monocyte adhesion.

## Materials and methods

### TMAO and animals

TMAO was purchased from Sigma (St. Louis, MO, U.S.A.). C57BL/6 mice (6–8-week-old males) were obtained from the animal house of Peking University, Beijing, China.

### Cell lines and cell culture

The human monocyte cell line THP-1 was purchased from Cell Resource Center, Institute of Basic Medical Sciences, Chinese Academy of Medical Sciences, Beijing, China. Cells were cultured in RPMI 1640 medium (HyClone, U.S.A.) containing 10% FBS. Human umbilical vein ECs (HUVECs) were isolated from umbilical veins [22]. The cells were cultured in extracellular matrix (ECM) (ScienCell, U.S.A.) containing 5% FBS, 1% EC growth supplement and 1% penicillin/streptomycin solution. The cells were then cultured in a humidified incubator with 5% CO_2_ at 37°C. HUVECs of passage 2–6 were used for experiments.

### Cell viability assay, lactate dehydrogenase releasing test and 5-bromo-2-deoxyuridine assay

For the MTT assay, HUVECs (5 × 10^3^ cells/well) were seeded in 96-well plates, cultured overnight and treated with varying concentrations of TMAO (0, 10, 50, 100 μmol/l) for 24 h. And then added 10 μl MTT solution to each well at a final concentration of 0.5 mg/ml and incubated for an additional 4 h. At the end of incubation, DMSO (150 μl) was added to each well and then the absorbance was measured at 570 nm by a microplate reader (Varioskan Flash, Thermo Fisher).

HUVECs were incubated with indicated concentrations of TMAO for 24 h, lactate dehydrogenase (LDH) activity in the culture media and cell lysates was respectively analysed using an LDH Assay Kit (Beyotime Institute of Biotechnology, China). Results were expressed as the percentage of LDH leakage, which was the ratio of LDH activity in the media to total LDH activity.

Cell proliferation was analysed using the 5-bromo-2-deoxyuridine (BrdU) assay. Briefly, equal numbers (5 × 10^3^ cells/well) of HUVECs were seeded in 96-well plates. Confluent HUVECs were then treated with TMAO (0, 10, 20, 40, 80, 100, and 200 μmol/l). Cell proliferation was measured for 48 h using BrdU assay kit according to the manufacturer’s protocol with stop solution (Roche Cell Proliferation ELISA BrdU colorimetric assay). The absorbance at 450 nm was measured within 5 min after adding the stop solution [23].

### Transwell migration assay

Quantificative migration assays with HUVECs were performed as described previously. In brief, the chambers with 8.0 µm of pore (Minicell, Millipore, U.S.A.) were put in 24-well plates, the lower chamber was added with 500 µl of complete medium and HUVECs (10^5^ cells/well) were suspended in 300 μl of serum-free medium containing indicated concentrations of TMAO (0, 10, 50, and 100 μmol/l) and then placed in the upper chamber. Cell migration was allowed to proceed for 24 h at 37°C in a 5% CO_2_ incubator. After incubation, the cells on the upper surface of the filter were removed by a soft cotton swab and the migrating cells were fixed with 4% paraformaldehyde, and stained using Crystal Violet (Beyotime, Nantong, China). Migration was assessed by photographing under an inverted microscope (Leica, Germany) and quantified by counting the number of stained cells from five random fields at 200× magnification [24].

### HUVEC-ECM adhesion assay

Cell adhesion was examined by the MTT assay as previously described. In brief, 96-well flat bottom plates were covered with 2 μg/well of basement membrane matrix (Matrigel, BD) for 1 h at 37°C, then blocked with 2% BSA for 2 h at 37°C followed by two washes. HUVECs seeded on a six-well plate were exposed with TMAO (0, 10, 50, and 100 μmol/l) for 24 h. After harvesting with trypsin-EDTA, the cells (10^5^ cells/well) were seeded on ECM-precoated 96-well plates and then incubated for 45 min at 37°C, after which the cells were washed twice with PBS to remove non-adherent cells. MTT colorimetric assays read at 490-nm wavelength were used to examine the absorbance of adherent cells. Six parallel wells were set up for each group [25,26].

### Measurement of adhesion molecules expression in HUVECs

Adhesion molecules expression was measured by immunocytochemistry. Briefly, HUVECs were plated in 96-well plates. Confluent HUVECs were serum starved for 6 h and treated with TMAO (0, 10, 50, and 100 μmol/l) for 6 h at 37°C, TNF-α was served as the positive control. Then, HUVECs were incubated with rabbit anti-ICAM-1 (PB0053, Boster) or rabbit anti-VCAM-1 (BA0406, Boster) or rabbit anti-E-selectin (BA0615, Boster) (1:200; Boster, China) in First Antibody Dilution Buffer for 2 h at 37°C. Omission of primary antibody was conducted in negative controls. And then the cells were incubated with a horseradish peroxidase-conjugated antibody (1:1000, Abcam, U.S.A.) for 1.5 h at 37°C. Quantification was performed by measuring the absorbance at 450 nm by a TMB peroxidase EIA substrate kit (Bio-Med Innovation, China) [25]. PKC inhibitor, staurosporine (2.5 nmol/l), was used at the beginning of the treatment.

### Wound healing assay

HUVECs were seeded in 12-well plates at a density of 8 × 10^4 ^ cells/well and cultured overnight to create a confluent monolayer, and then created a cleared wound area by manually scraping with a 200-μl pipette tip. Cells were then incubated with the indicated concentrations of TMAO (0, 10, 50, 100 μmol/l) for 24 h at 37°C. Cells were fixed with methanol and then stained with Crystal Violet, and the wound-healing degree was photographed under an inverted microscope (Leica). Cells that migrated into the gap were counted in seven random high power (100×) fields [25].

### *In vitro* adhesion assay

In brief, confluent HUVECs on 96-well plates were starved for 6 h and treated with TMAO (0, 10, 50, and 100 μmol/l) for 6 h at 37°C. Thereafter, cells were exposed to human THP-1 monocytes (10^5 ^cells/well) for 40 min. Non-adherent THP-1 cells were removed by washing one time with PBS, the OD (optical density) value at 450 nm was measured. Six parallel wells were set up for each group. To ensure high-quality digital photographs, THP-1 cells were pre-stained with Hoechst 33258 (HARVEY, Beijing, China), and adherent cells were counted in randomly selected optical fields taken from an inverted microscope (Leica). Neutralizing mAb and the PKC inhibitor, staurosporine (2.5 nmol/l), were used at the beginning of treatment [27].

### PKC activity assay

The PKC activity in the HUVEC lysates was determined by PepTag® Non-Radioactive Protein Kinase Assays (Promega, V5330, U.S.A.). As described in the manufacturer’s instructions, 5 × 10^6 ^cells were removed to prepare PKC extracts. The brightly coloured, fluorescent peptide substrate was specially phosphorylated by PKC, and its net charge was altered from +1 to −1. This change in the net charge of the substrate allowed the phosphorylated and non-phosphorylated versions of the substrate to be rapidly separated on an agarose gel. [25].

### Immunoblotting

BCA protein assay kit was purchased from Thermo Fisher Scientific (U.S.A.). Anti-p-NF-κB p65 (CST, Catalogue number #3303) and secondary antibodies were purchased from Cell Signaling Technology (U.S.A.). Details of immunoblotting have been described elsewhere.[28]

### Nuclear extract preparation

Nuclear proteins were extracted following the instructions for NE-PER Nuclear and Cytoplasmic Extraction Reagents (Thermo Fisher Scientific, #78833).

### Immunohistochemistry

Histology tissues were fixed in 4% paraformaldehyde and subsequently embedded in paraffin wax. Six-micrometre thick sections were cut from each paraffin-embedded tissue and collected on microscope slides and then dewaxed with xylene and rehydrated with ddH_2_O. Endogenous peroxidases were blocked by 0.3% H_2_O_2_ solution (diluted with methanol) for 12 min. Antigen retrieval was conducted in EDTA working solution (10 mmol/l, pH 8.0) for 10 min at 92°C. The tissue sections were blocked by 5% goat serum for 1.5 h at 37°C, after which sections were incubated with primary antibodies (rabbit anti-ICAM-1 (PB0054, Boster), VCAM-1 (BA0406, Boster) or E-selectin (BA0615, Boster); dilution 1:200) overnight at 4°C. The tissue sections were then treated with appropriate HRP-conjugated secondary antibodies for 40 min at 37°C and antigen–antibody reactions were stained with 3,3-diaminobenzidine. The adhesion molecules expression was examined with a Nikon Eclipse Ti microscope under high power (400×) fields. Adhesion molecules expression was quantified by Leica Q550CW image analysis system.

### p-NF-κB staining

HUVECs on coverslips were starved for 4 h and treated with TMAO (0, 10, 50 and 100 μmol/l) for 6 h at 37°C. And then HUVECs were fixed with 4% paraformaldehyde, after which blocked by 10% goat serum for 1.5 h at 37°C. For p-NF-κB fluorescent staining, the coverslips were first incubated with the antibodies rabbit anti-p-NF-κB (1:200) and then the secondary goat anti-rabbit IgG/PE antibody (1:200) (Bioss, Beijing). At last, the coverslips were incubated with a reagent containing DAPI (Sigma, U.S.A.) for 10 min and mounted on slides. Fluorescence was detected by confocal laser scanning microscopy (Leica, Germany).

### *Ex vivo* adhesion assay

For *ex vivo* adhesion experiments, 100 μl PBS and 100 μl various high concentrations of TMAO were respectively given by tail vein injection, which makes the drug concentration in whole blood reach to final concentrations (0, 0.1, 1 and 10 mmol/l). Twenty-four hours later, mice were anaesthetized with ketamine and 5% chloral hydrate. Under sterile conditions, the heart was exposed through a left thoracotomy, and perfused from the left ventricle with normal saline until the blood was washed out. Then, Hoechst-labelled THP-1 monocytes (1 × 10^7^ cells/ml) were perfused from the left ventricle to the aorta and incubated for 45 min at 37°C. Non-adherent THP-1 cells were removed by perfusion with normal saline. Aortas were harvested at the level of the aortic arch to the abdominal aorta beyond renal arteries and subsequently fixed in 4% paraformaldehyde solution. Adhesion was observed by confocal laser scanning microscope (Leica, Germany) and quantified by calculating the areas of fluorescent monocytes attached to the vascular surface.

### Statistical analysis

Statistical analysis was carried out using a one way ANOVA with Tukey’s post-test; *P*<0.05 was considered significant. Error bars represent mean ± S.D.

## Results

### Cell viability of HUVECs undergoing TMAO treatment

We firstly investigated the effect of TMAO on cell viability. We found that there was no difference in cell viability as determined using both the MTT assay (Figure 1A) and LDH release test (Figure 1B).

**Figure 1:** The effect of TMAO on cell viability HUVECs were exposed to different TMAO levels (0, 10, 50 and 100 μmol/l) for 24 h, cell toxicity assay was tested by MTT assay (**A**) and LDH assay test (**B**). Results are presented as the mean ± S.D. of three independent experiments.

### Self-repair capacity of HUVECs was reduced by TMAO

Atherosclerotic CVD is initiated by vascular EC injury, which is frequently linked with endothelial dysfunction [29]. We observed significantly decreased vascular self-repair capacity of HUVECs treated with TMAO.

To explore the influence of TMAO on cell proliferation, colorimetric BrdU assay were conducted on HUVECs treated with varying doses (0–200 μmol/l) of TMAO for a 48-h period. The cells exhibited a dose-dependent reduction in proliferation and showed 0.76 ± 0.23 fold reduction with TMAO treatment (100 μmol/l) at 48 h compared with control, as reflected by the decreasing absorbance (Figure 2A).

**Figure 2:** Self-repair capacity of TMAO-treated HUVECs (**A**) HUVECs were treated with different doses of TMAO (0, 10, 20, 40, 80, 100 and 200 μmol/l) for 48 h. Relative cell proliferation was examined by BrdU ELISA and expressed as fold of TMAO-treated cells compared with control. (**B**) HUVECs were exposed to different TMAO levels (0, 10, 50 and 100 μmol/l) for 24 h, TMAO-stimulated HUVECs attached to ECM was measured, *n*=3. (**C**, **E**) HUVECs were incubated with TMAO at the indicated concentrations in the upper chamber for 24 h. Transwell assay was used to determine the cell migration and pictures were shown in high power (200×). Cell migration was quantified by cell counting. (**D**, **F**) Monolayer HUVECs were wounded by manual scraping and incubated with TMAO at the indicated concentrations for 24 h and then photographed in high power (100×). Cells migrating into the gaps were quantified by cell counting. Results are presented as the mean ± S.D. of three independent experiments; (*P<0.05, **P<0.01, ***P<0.001).

We secondly determined the effect of TMAO on HUVEC-ECM adhesion. The results showed a dose-dependent reduction in HUVEC-ECM adhesion, which was reduced by 0.92 ± 0.08 fold compared with control following 100 μmol/l of TMAO treatment (Figure 2B). Moreover, HUVECs migration was inhibited by TMAO in both wound healing assay and transwell migration assay and all the effects were dose-dependent. As shown in Figure 2C,E, the number of cells that migrated through the polycarbonate membrane was decreased from 175.10 ± 23.70 to 106.90 ± 8.04. As shown in Figure 2D,F, the amount of HUVECs that migrated into the gaps was reduced from 232.2 ± 38.11 to 175.9 ± 55.59.

### TMAO promotes monocyte adhesion to HUVECs via positively regulating VCAM-1 expression

Monocyte adhesion is a key process in the pathogenesis of atherosclerosis. To uncover the effect of TMAO on monocyte adhesion to HUVECs, HUVECs were treated with various doses of TMAO for 6 h and co-cultured with THP-1 cells for an additional 40 min. Adhesion of THP-1 cells to HUVECs was stimulated by TMAO in a dose-dependent manner as the amount of adherent THP-1 cells increased from 0.99 ± 0.15 to 1.25 ± 0.32 (Figure 3A,B).

**Figure 3:** THP-1 cells adherence to HUVECs induced by TMAO is attributed to VCAM-1 up-regulation (**A**, **B**) HUVECs were starved for 6 h and treated with TMAO (0, 10, 50 and 100 μmol/l) for 6 h. Images represent the mean of adherent monocytes per microscopic field. Scale bar =50 μm. The results were normalized to the number of control cells. (**C**) HUVECs were treated with TMAO at the indicated concentrations as above for 6 h. VCAM-1, ICAM-1 and E-selectin expression in HUVECs were examined by cell ELISA. Results are represented as fold of TMAO-treated cells in comparison with control. (**D**) HUVECs were incubated with no antibody, negative control antibody and anti-VCAM-1 antibody for 30 min at 37°C before the adhesion assay, the fold change is showed. The results are presented as the mean ± S.D. of three or more independent experiments; (*P<0.05, **P<0.01).

During the process of cell adhesion, cell adhesion molecules most likely play an important role in cell communication [16,30,31]. The cell ELISA results suggested that treatment of TMAO up-regulated VCAM-1, but not ICAM-1 and E-selectin. When HUVECs were treated with 100 μmol/l of TMAO, expression of VCAM-1 reached 1.20 ± 0.17 fold increase compared with control (Figure 3C). In addition, blocking antibody to VCAM-1 was used to confirm the roles of VCAM-1 in the adhesion of THP-1 cells to HUVECs. Adhesion of THP-1 cells to HUVECs was decreased from 1.207 ± 0.219 to 1.033 ± 0.132 in the presence of anti-VCAM-1 antibody (Figure 3D).

### TMAO promotesTHP-1 adhesion to mice aortic wall and increases VCAM-1 expression in mice aortic ECs

To further confirm the contribution of TMAO-induced VCAM-1 expression on monocyte adhesion *ex vivo*, we performed adhesion assays with aorta isolated from C57BL/6 mouse. Treatment with TMAO significantly increased monocytes adhesion to the aorta of C57BL/6 mice (11.39 ± 3.57 fold change, 1 mmol/l treatment compared with 0 mmol/l treatment; 21.58 ± 10.51 fold change, 10 mmol/l treatment compared with 0 mmol/l treatment) (Figure 4A,E) and VCAM-1 expression (1.14 ± 0.09 fold change, 1 mmol/l treatment compared with 0 mmol/l treatment; 1.18 ± 0.07 fold change, 10 mmol/l treatment compared with 0 mmol/l treatment) (Figure 4B,F). However, no change was observed in the expression of ICAM-1 and E-selectin compared with control (Figure 4C,D,F).

**Figure 4:** TMAO injection promotes THP-1 adhesion to the aortic wall and increases VCAM-1 expression (**A**) TMAO treatment increased THP-1 cell adhesion to the aorta vascular wall. Results were shown as fluorescence in confocal microscopic images. Scale bars =250 μm. Images represent the immunohistochemical staining of VCAM-1 (**B**), ICAM-1 (**C**) and E-selectin (**D**) in mice aorta vascular ECs. Arrows in (B) represent VCAM-1-positive areas. Scale bars =50 µm, (*n*=4). (**E**) Quantification of adhesion on aorta, the result was expressed as areas of monocytes attached to aorta. Data are expressed as mean ± S.D. (**F**) Quantification of adhesion molecules expression, the fold change is presented as mean ± S.D.; (*P<0.05, **P<0.01, ***P<0.001).

### TMAO activated NF-κB in HUVECs

Activation of NF-κB was suggested to be essential and sufficient for endothelial adhesion molecules expression in ECs. Coincidently, in our study, the cellular protein level of p-NF-κB was increased from 0.98 ± 0.17 to 1.39 ± 0.16 (Figure 5A,B). To confirm the effect of TMAO on NF-κB, we next detect p-NF-κB by immunofluorescence technique. We found that treatment with TMAO resulted in phosphorylation of NF-κB (red fluorescence) and enhanced p-NF-κB aggregation and localization to nucleus in dose-dependent manner (Figure 5C).

**Figure 5:** TMAO activated NF-κB in HUVECs HUVECs were treated with TMAO (0, 10, 50 and 100 μmol/l) for 6 h in serum-free media. (**A**) Effect of TMAO on the protein level of p-NF-κB was determined by Western blot. p-NF-κB relative expression ratios were determined by grey-scale image analysis. (**B**) Results are presented as the mean ± S.D. of six independent experiments, (*P<0.05, **P<0.01). (**C**) p-NF-κB was also detected by fluorescent staining (red fluorescence) in HUVECs on coverslips. Blue fluorescence represented nucleus. Fluorescent images were detected by confocal laser scanning microscopy. Scale bars =25 µm.

### TMAO-induced endothelial dysfunction is associated with PKC activiation

It has been known that the activity of PKC plays an important role in regulating endothelial dysfunction, including inflammation and adhesion [27]. PKC activity was examined in HUVECs treated with TMAO. In the present study, TMAO elevated PKC activity compared with control in a dose-dependent manner (Figure 6A). Interestingly, treatment with staurosporine inhibited NF-κB phosphorylation (Figure 6B). Moreover, staurosporine treatment significantly diminished the increased VCAM-1 expression and THP-1-HUVECs by TMAO (76.9% decrease and 86.2% decrease respectively) (Figure 6C,D). These data indicated that the activation of PKC was at least in part responsible for TMAO-induced endothelial dysfunction.

**Figure 6:** TMAO activated NF-κB in HUVECs TMAO-induced endothelial dysfunction is associated with PKC activiation (**A**) HUVECs were treated with TMAO (0, 10, 50 and 100 μmol/l) for 6 h in serum-free media. Cell lysates from TMAO-treated cells were analysed by the PepTag non-radioactive PKC assay. HUVECs were treated with 100 μmol/l TMAO in the presence or absence of staurosporine (2.5 nmol/l) for 6 h and then p-NF-κB expression (**B**), VCAM-1 expression (**D**) and monocyte adhesion to HUVECs (**E**) were measured. The results are presented as the mean ± S.D. of three or more independent experiments (*P<0.05, **P<0.01).

## Discussion

Several clinical and metabolic studies have demonstrated that elevated concentration of plasma TMAO can be a CVD risk independent of traditional risk factors [32]. Multiple studies have been done to explore the mechanism by which high plasma level of TMAO may cause the acceleration of atherosclerotic CVD. These studies showed that: (1) TMAO may modulate cholesterol and sterol metabolism [33 ]; (2) TMAO could cause low glomerular filtration rate [34] and impair glucose tolerance [35 ]; (3) TMAO could also increase arterial blood pressure [36]. They are all independent risk factors for CVDs. However, the molecular mechanisms underlying the effects of TMAO on monocyte–EC interaction remain unclear. While we were preparing this manuscript, Seldin et al. [37] reported that TMAO promoted vascular inflammation through signalling of mitogen-activated protein kinase and nuclear factor-κB. Altogether, our data explored the likely mechanism of TMAO-induced atherogenesis. In the present study, we reported a novel role of TMAO as a regulator of endothelial dysfunction and an inducer of monocyte recruitment during atherosclerosis.

Endothelial damage and monocyte adhesion are critical events in the initiation of atherosclerosis [29,30]. EC proliferation and migration may play a crucial role in vascular self-repair [28]. EC monolayer integrity is maintained by the replacement of damaged cells via proliferation and migration of neighbouring cells [38]. The present study suggested that TMAO inhibited HUVEC proliferation (Figure 2A) and adhesion to the ECM (Figure 2B). Moreover, TMAO markedly suppressed EC migration in both the transwell migration assay (Figure 2C,E) and the wound healing assay (Figure 2D,F) in a dose-dependent manner. These results indicated that elevated plasma TMAO inhibited the capacity of vascular self-repair. Previous studies demonstrated that animal diet supplemented with TMAO resulted in enhanced levels of SR-A1 and CD36 in macrophages and endogenous formation of foam cells [6]. Consistent with this finding, the present study suggested that TMAO positively regulated VCAM-1 expression in ECs (Figures 3C and 4B), leading to increased monocyte adhesion (Figures 3A,B and 4A), which are the early cellular hallmarks of the foam cell formation, in both *in vitro* and *ex vivo* experiments.

Vascular inflammation is a basic pathological mechanism of atherosclerosis. The increased expression of cellular adhesion molecules, such as VCAM-1 and ICAM-1, plays an important role in endothelial dysfunction and is essential to recruiting monocytes from the circulation. PKC activation up-regulates adhesion molecules in ECs [27]. Four PKC isoforms have been identified in human ECs, namely PKC-α, PKC-δ, PKC-ε and PKC-ζ [16]. Although the present study did not explore the roles of different PKC isoforms in TMAO-treated ECs, we showed that total PKCs activity was increased in TMAO-treated ECs (Figure 6A). It has been shown that the NF-κB activation pathway is initiated by various PKCs [39]. Coincidently, we found that TMAO promoted NF-κB phosphorylation (Figure 5). p-NF-κB enters the nucleus to regulate genes expression. Inducible genes, including IL-1β, IL-6, IL-8, tumour necrosis factor-α, monocyte chemotactic protein-1, cyclooxygenase-2, VCAM-1 and ICAM-1 are known to be activated by NF-κB. In the pathology of atherosclerosis, NF-κB activation is believed to underlie the regulated expression of VCAM-1 [40]. In the present study, VCAM-1 expression and monocyte adhesion were increased both in TMAO-treated cells (Figure 3) and TMAO-treated artery (Figure 4) compared with control. Moreover, increased VCAM-1 expression and monocyte adhesion were significantly diminished by VCAM-1 neutralizing antibody and PKC inhibitor (Figures 3D and 6). Therefore, we speculate that TMAO may function as a positive upstream regulator of PKC/p-NF-κB signalling and indirectly activates the VCAM-1 promoters and promotes monocyte adhesion. As shown in our results, PKC inhibition did not completely abolish VCAM-1 expression and monocyte adhesion stimulated by TMAO, indicating that other signal pathway may potentially contribute to the effects of TMAO on monocyte adhesion. Another important question is: how TMAO affects cellular signal transduction, through selective recepter or other ways? It has been reported that TMAO can serve as a small chemical chaperone, influencing the structure and function of some proteins [41,42]. We assume that TMAO is uptake into cells and subsequently combines with PKC activator such as PIP2, syndecan-4 etc. [43], and together they participate in the activation of PKC. However, further research is needed (Figure 7).

**Figure 7:** The likely molecular mechanism of TMAO-induced monocyte adhesion This pathway suggests that TMAO affects vascular endothelial ECs and subsequently stimulates activation of PKC. Then, NF-κB is activated by phosphorylation and translocates to the nucleus. NF-κB activation induces VCAM-1 expression and monocyte adhesion to the vascular wall.

In conclusion, data presented here show that TMAO is a novel positive regulator of endothelial dysfunction and the effect of TMAO on endothelial dysfunction is partly attributable to activation of PKC/NF-κB, leading to elevated expression of VCAM-1 and monocyte adhesion. Although the receptor for TMAO has not yet been identified, the exploration of exact mechanism can lay the foundation for targeted atherosclerosis therapy.

## Abbreviations

BrdU: 5-bromo-2-deoxyuridine
CVD: cardiovascular disease
EC: endothelial cell
ECM: extracellular matrix
HUVEC: human umbilical vein EC
ICAM-1: intercellular adhesion molecule-1
IL: interleukin
LDH: lactate dehydrogenase
NF-κB: nuclear factor-κB
PIP2: phosphatidylinositol 4,5-bisphosphate
PKC: protein kinase C
TMAO: trimethylamine N-oxide
VCAM-1: vascular cell adhesion molecule-1
